# Research on the Transformation from Financial Accounting to Management Accounting Based on Drools Rule Engine

**DOI:** 10.1155/2022/9445776

**Published:** 2022-04-20

**Authors:** Rui Liu, Yuqin Wang, Jing Zou

**Affiliations:** ^1^School of Accounting, Wuhan College, Wuhan 430212, Hubei, China; ^2^The Centre of Finance Research, Wuhan University, Wuhan 430212, Hubei, China

## Abstract

With the development of Internet economy and the advent of artificial intelligence era, the transformation from financial accounting to management accounting has become an inevitable trend of financial management among companies. In this paper, the significance of the transformation from financial accounting to management accounting is expounded under the background of artificial intelligence, and the current situation, problems and reasons of the transition are analyzed. In addition, the development of self-management accounting system based on Drools rule engine is put forward, including rule management, rule engine and so on. The core processes such as pattern matching and auto-billing are analyzed, and then the core subsystems such as data receiving and processing, accounting rule engine are designed in detail. Finally, the technological advancement and structural stability of this system are discussed, which can provide reference for promoting the transformation from financial accounting to management accounting under artificial intelligence.

## 1. Introduction

The deep combination of artificial intelligence and financial management has promoted the development of financial management among enterprises towards automation and intelligence. Under this trend, traditional financial methods have been difficult to apply to modern financial management. Financial management must undergo subversive changes to fully adapt to the development of artificial intelligence [1]. Under the background of artificial intelligence, financial management needs to actively use information technology, integrate financial data, and provide guarantee for various business management decisions of enterprises, so as to avoid the lag of traditional financial management. Considering the current situation, with the help of a new generation of scientific and technological revolution and industrial transformation, artificial intelligence has achieved good application in many professional fields. Combined with relevant survey [2], in the next 10 years, the accounting industry will probably be the professional field most affected by the application of artificial intelligence. From the perspective of accounting management, the concept of traditional financial accounting management has been weakened by the management accounting, and the repetitive labors in financial work can be reduced by combining the artificial intelligence, which ensures the improvement of financial quality [3–5]. It is not difficult to see that with the support of artificial intelligence technology, the transformation and development from financial accounting to management accounting will be further promoted.

With the rapid development of information technology and the global popularity of artificial intelligence, the management accounting system has gone through a process from manual accounting to computerized accounting to informatization. After entering the twenty-first century, under the impact of the rapid development of artificial intelligence and e-commerce, the emergence and development of accounting information system has been regarded as the inevitable trend [6]. Network accounting information system is based on Internet technology, which reflects the accounting and supervision of financial resources within the whole enterprise, which realizes comprehensive, timely and dynamic accounting supervision, prediction and management of the whole enterprise [7]. By providing enterprises with accounting methods and financial management modes under the network environment, accounting management is gradually becoming standardized, and the supervision and accounting functions of accounting are fully exerted. Therefore, Promoting the informatization, networking and automation of management accounting system in the era of artificial intelligence is helpful to the transformation from traditional financial accounting to management accounting, which has become the new direction of development in accounting system.

## 2. Analysis of Financial Accounting and Management Accounting under Artificial Intelligence

### 2.1. Definition of Financial Accounting and Management Accounting

#### 2.1.1. Financial Accounting

The so-called financial accounting refers to the general term of economic management activities for investors and creditors who have economic interested relationship with the development of enterprises outside the enterprise and information about financial status and profitability provided by relevant government departments [8, 9]. In the development of modern enterprise, financial accounting is one of the most important management items. Generally speaking, through a series of financial accounting procedures, financial management can provide useful decision-making information for managers, and can promote enterprises to run efficiently in the process of serving the market economy.

#### 2.1.2. Management Accounting

The so-called management accounting refers to a branch of accounting [10, 11] which is separated from traditional accounting, integrates accounting and financial management, and focuses on providing economic forecast, investment decision-making, management improvement and economic benefit service for enterprise managers. Theoretically, the concept of management accounting enriches the related research on accounting and management in academic circles. From the practical function point of view, where management accounting mainly has the following functions: first, it can put forward objective and practical suggestions on the development of enterprises based on data from the financial point of view, so that the development of enterprises can be more scientific and reasonable; Second, it is able to grasp the capital status of an enterprise in the process of development in time, which makes the context of the enterprise's capital clear; Third, to a certain extent, it can reduce the cost in the process of business operation and expand the profits of enterprises. At the same time, it can also make full preparations for further investment to a certain extent, and ensure the steady progress of enterprises.

### 2.2. Differences between Financial Accounting and Management Accounting

In recent years, with the rapid development of artificial intelligence technology, management accounting system has been successfully integrated into various professional fields for practical application, and achieved remarkable results. For financial management, with the support of decision-making of artificial intelligence technology, the differences between financial accounting and management accounting are becoming more and more obvious [12].

On the one hand, under the background of “artificial intelligence,” the financial accounting work of enterprises is more focused on serving the management of enterprises. Generally speaking, in the process of business management, enterprises will involve a large number of capital transactions and financial data. If only the previous financial accounting methods are used for management, in terms of financial integration, it is easy to make mistakes. By using informatization management, enterprise financial data information can be integrated and given feedback to managers in the form of financial statements, which can effectively reduce errors of management [13]. At the same time, in the management of economic activities, the financial department of an enterprise can complete the decision-making analysis of financial data by means of management accounting, in which managers can make forward-looking deployment for the direction in a certain period according to the information data fed back by the financial report [14].

On the other hand, the methods of financial management become more flexible and diverse. Compared with the traditional financial management model, the financial accounting of modern enterprises pays more attention to reflecting the diversified characteristics, requiring financial managers to flexibly adjust the selected management methods according to the actual operation of enterprises. The essential purpose of financial accounting and management accounting is to realize high-quality process of financial management, but there are still some differences in responsibility [15]. For example, financial accounting reports are more strict in preparation than management accounting, and legal responsibility is also relatively strict. In other words, Accounting is more obvious in terms of financial constraint, while management accounting can actively combine artificial intelligence and other technical contents to realize systematic treatment of financial management, and timely adjust financial management according to the financial operation, with more obvious decision-making characteristics.

### 2.3. Problems in the Current Management Accounting System

In order to promote the transformation from financial accounting to management accounting, first, the current management accounting system must be optimized. At present, the management accounting system used by most companies is a software system under computerized accounting. The whole process of the traditional management accounting system is: transaction, voucher, accounting, reconciliation, trial calculation, financial statements, most of which need manual participation, thus exposing some urgent problems [16–19].

#### 2.3.1. Inefficient Manual Accounting

The basic function of accounting is calculation and supervision, so in the daily business of the company, every transaction involving capital changes needs accounting. From the traditional cycle process, it can be seen that from the transaction to the voucher accounting, reconciliation, trial calculation, and the issuance of financial statements, manual intervention is needed because it is mainly designed for traditional invoicing enterprises, while the turnover rate of inventory funds in traditional enterprises is slow, so it has no need for real-time auto-billing. However, with the in-depth development of artificial intelligence, the Internet-based financial enterprise does not have the concept of inventory, but provides online payment or financial services, with rapid transactions. Therefore, their capital turnover rate is fast, and manual accounting is obviously inefficient and cannot meet the actual business needs of the company's financial management.

#### 2.3.2. Low Accuracy Rate of Data

The current management accounting system cannot reflect the detailed changes of the whole business or individual business of the company. The data recorded by accountants are generally the data after statistics of various business systems, due to the changes of transaction data in real time. Moreover, the financial personnel can only record the total statistics of each business system in advance, so the changes of individual transactions cannot be reflected in the current financial system, and all the business systems are connected to the management accounting system.

#### 2.3.3. Nonnetworking Based on Single Machine

At present, the company's management accounting system is based on the client stand-alone mode, and the financial personnel need to install the client first. Without the client's personal PC or mobile devices such as mobile phones and IPAD, the financial personnel cannot count the financial statements, and managers cannot analyze and make decisions according to the financial statements. In addition, the management accounting system under computerized accounting is not based on the Internet. Under the circumstance that enterprises are constantly building various information systems, it will be out of touch with the major information systems of enterprises. For example, the data format of each business information system will be inconsistent with the format required by the management accounting system. Therefore, the computerized accounting software based on single machine can easily lead to the formation of information islands.

## 3. Design and Implementation of Management Accounting System Based on Drools

Management accounting system is undoubtedly very important during the normal operation of management activity. It can help managers to know the profit and loss situation of enterprises in time, so as to formulate reasonable strategies. From the above analysis, it can be seen that in order to promote the transformation from traditional financial accounting to management accounting, first of all, it is necessary to solve the problems that the current accounting management system needs to manually record the accounting vouchers of each transaction, as well as it cannot provide business rules to automatically match transaction orders with large amounts of data, and cannot automatically make trial balance [20]. Therefore, a management accounting system based on Drools rule engine is designed in this paper, *s* as to better realize the faster and better transformation of financial accounting.

### 3.1. Introduction of Drools Rule Engine Technology

#### 3.1.1. Basic Concepts of Rule Engine

Drools is a popular rule engine component at present, while its basic components include business rules and rule engines are. Here, the definition, composition and workflow of rule engines are briefly introduced.

Definition of business rules: in essence, business rules can also be understood as a set of conditions and operations, which include conditions and actions. When a business fact meet certain conditions, certain actions will be executed, which is similar to the meaning expressed by conditional statements if…then… in program [21]. The rules files of this system are managed by Drools Guvnor.

Definition of rule engine: rule engine is the environment where rules are to be executed. Its main functions contain describing rules, compiling rules, rule execution and resolution of rules conflict, which is an independent component that can be embedded into programs [22]. At present, the rule engines of comparative processes are: Drools of Jboss Company of the United States, VisualRules of Qizheng Company of China and ILOG of IBM abroad.

Composition and workflow of rule engine: “How to make computers think like humans?” This is a problem in the field of Artificial Intelligence, which includes [23, 24]: Neural Networks, Genetic Algorithms, Decision Trees, Frame Systems and Expert Systems. Rule engine is one of Expert Systems, which is also known as knowledge-based system. It is a system based on rule base, transferring facts and drawing conclusions. The structure of the rule engine is shown in Figure 1:

It can be seen from the figure that the rule engine consists of three parts [25]: Production Memo, Working Memory, and inference Engine, while the inference engine consists of Pattern Macher, Agenda, and is also known as Conflict Resolution. When one or more facts are met by multiple rules, conflicts will occur. At this time, the Agenda is responsible for coordinating the execution sequence of Activations. Each activation consists of a rule and a fact or multiple facts. The Execution Engine is responsible for executing the rules selected by the Agenda. The actions triggered by the rules may produce new facts, which will be readded to the Working Memoir fact base.

#### 3.1.2. Matching Algorithm of Rete Pattern

Drools is an open source rule engine that coded in Java, and adopts Rete algorithm to calculate rules [26]. The implementation of DroolsRete is called ReteOO which means that Drools has enhanced and optimized the implementation of Rete algorithm of object-oriented system. Drools allows users to express rules of business logic declaratively. Rules in non-xml native language can be coded which is easy to learn and understand [27] and Java can be embed directly into the rules file. In addition, Drools has other advantages:

1. Supported by an active community
2. Convenient to use
3. Fast execution
4. More and more popular among Java developers
5. Comply with Java rule engine API(JSR94)
6. Free

Drools uses a rule-based method to implement an expert system. It is more accurately classified as a production rule system [28]. The production rule system is Turing complete, focuses on knowledge representation, and expresses propositions and first-order logic in a concise and nonfuzzy way. The brain of the production rule system is an inference engine Figure 2. It can be extended to numerous rules and fact reasoning engines to match facts and data according to production rules (also known as production rules or fair rules) to infer the conclusions that lead to actions.

### 3.2. Design of Systematic Architecture

By analyzing and explaining the Drools rule engine based management accounting system, the network architecture, system software architecture and other aspects are analyzes and compared with similar systematic architectures which illustrates the technical advantages of implement based on Drools rule engine.

#### 3.2.1. Systematic Network Architecture

The management accounting system is a comprehensive application system with a large scale of data. The design of platform system should fully consider the needs of the actual accounting business, and on this basis, determine the overall goal of the system, so that the system has the characteristics of advanced practicality, high performance, security, scalability and excellent compatibility [29]. The network architecture of the management accounting system is shown in Figure 3.

B/S (Bowser/Server) architecture is adopted where the client does not need to be installed, and users only need to pass the comparison on personal computers, laptops and IPAD, then Internet browsers such as Rome and Safari can realize the interaction with the management accounting system [30]. First, users initiate online transactions to the company's business system through HTTP/TCP requests. Besides recording data in the databases of their respective systems, at the same time, the ActiveMQ message is sent to ApacheActiveMQ server through TCP/IP protocol, the data receiving and processing subsystem reads the message of ActiveMQ server through TCP/IP protocol, and then calls the interface of rule engine subsystem through Netty communication framework of TCP/UDP protocol. Afterwards, the data receiving and processing subsystem converts the transaction message into accounting voucher and then the accounting voucher is sent to the rule engine subsystem for processing. After receiving the accounting voucher object, the rule engine subsystem converts the accounting voucher into the corresponding accounting record according to the predefined accounting rules.

The other way is completed by the batch processing task of the data receiving and processing subsystem, because each business system needs to access the management accounting system step by step for a period of time, and at the same time, it is necessary to keep an account of the historical transaction data of each business system, so the accounting batch processing is needed to process the batch processing task through ORACLE's DB1ink technology, so as to let the database of the management accounting system be directly connected to the database reserve of each business system.

#### 3.2.2. Systematic Software Architecture

In the design process, the mainstream three-tier architecture system is adopted, and the whole architecture system is divided into data access layer, business logic layer and presentation layer, which makes the software design convenient for modularization and standardization, and is conducive to the development, maintenance and future expansion and upgrading of the system. The software architecture of management accounting system is shown in Figure 4.

1. Performance layer: it is provided for external end users, and is used by internal staff through the entrance of interoperation with major business systems. For example, it is provided for financial personnel with the back-office management subsystem of management accounting system. After the back-office management personnel log in to the subsystem, audit accounts, bank gateway, bank rate, query and report, etc will be set up. This layer is all displayed in the way of web browser, and users can use the most common browsers without installing any client program, which brings convenience to them.
2. Business logic layer: the main business logic of the management accounting system can be realized at this layer, which is mainly composed of four main subsystems: rule management subsystem, data receiving and processing subsystem, rule engine subsystem and accounting background management subsystem. At the same time, the short message system and mail system is externally connected. After the system error or some business is completed, For example, the data receiving and processing subsystem generates all the transaction data into accounting vouchers and accounting records, short messages and emails will be used to inform relevant developers and financial personnel. In addition, relevant data in Memocached cache system can be selected in order to optimize system performance, and ApacheActiveMq message queue system is used to receive transaction data messages of major business systems.
3. Data access layer: the business logic layer is connected to the data access layer through JDBC. This system uses the relational database Oraclel0g, and manages the basic data of the accounting system, such as basic data used in accounting rules, accounting subjects, bank gateway, bank rates, etc. Because it involves confidential data of company transactions, the production data is not allowed to be accessed by the test environment. At the same time, The release of DDL and DML in the database only allows special DBA to query and export related statements such as balance sheet, income statement, cash flow statement, etc., and is restricted to financial personnel and company management. The company's business system and management accounting system take Oraclel0g, where DBlink technology can be used to realize high-speed access between business system and accounting management system database.

The business module has been independent, and loose coupling is realized at the code level. Therefore, when adding or modifying accounting rules, there is no need to recompile the code and release a new system version, just edit the xml or drl rule file online, and all subsystems can adopt the Saturn framework developed by the company. The architecture of framework is clear and easy to maintain and expand, which has superior performance. Saturn framework is shown in Figure 5.

### 3.3. Systematic Implementation

#### 3.3.1. Implementation of Rule Management Subsystem

The main function of DroolsGuvnor rule management subsystem is to manage the rule files used by the rule engine subsystem, and to create and edit the rule files, check the grammar correctness, test and publish the rules.

Add repository: after the new repository is added, the role of the repository is to store rule file items. Click Authoring Administ Rational, then click Newreposito to add a new repository, and then fill it down step by step. Enter the name of the repository and the organizational unit to which it belongs. The relative location of the repository is git://localhost: 9418/AccountRepository. The version of the project file is controlled by git tool.

Add items: after the repository is created, create the Project of Drools rule file, and enter the description such as Project Name, Project Description, GroupID, ArtifactID, VersionID, etc. to create the rule file management project of the management accounting system.

Create a new data model:

after the project is created, it needs to create a data model, that is, the Fact model in the rule engine, which is created by DataModeler under the tools menu. Fill in the name of the model and the name of the package where it is located, then add the field name and field type for the new object type, and then click “Save” to save the object model.

Create a rule file: after the relevant data model is created, continue to create the rule file, and send it to create the rule file through the DRLfile in the NewItem, or through the GuideRule or GuideRuleTemplate option.

#### 3.3.2. Implementation of Rule Engine Subsystem

This system uses Maven technology to manage the dependency and construction. The project dependency on DroolsExpert [31]is configured in the root pom xml of the project as follows:

- <dependencies>⃞⃞
- <dependency>⃞⃞
- <groupld>org.drools</groupId>⃞⃞
- <artifactld>drools-core</artifactId>⃞⃞
- <version>5.5.0.FinaK/version)□⃞
- </dependency>⃞⃞
- <dependency>⃞⃞
- <groupId>org.drools</groupld>⃞⃞
- <artifactId>drools-compiIer</artifactId>⃞⃞
- <version>5.5.0.FinaK/version)□⃞
- </dependency>⃞⃞
- <dependency>⃞⃞
- <groupId>com.thoughtworks.xstream</groupId>⃞⃞
- <artifactld>xstream</artifactid)□⃞
- <version>l.3.1/version>⃞⃞
- </dependency>⃞⃞
- </dependencies>⃞⃞

#### 3.3.3. Implementation of Data Receiving and Processing Subsystem

The main function of the data receiving and processing subsystem is to receive the order transaction data of major business systems, convert the transaction data into accounting vouchers, and then call the rule engine subsystem to record the accounting vouchers into the management accounting system database. At the same time, there are two ways for data receiving and processing subsystem to receive data: single transaction and batch transaction.

The first way is to provide ApacheActiveMQ message queue address. Every transaction with cash in online business system will send a message to ApacheActiveX queue in real time. Then, the consumer asynchronously extracts the message, after extracting the transaction order data message, the data in JS0N string format are converted into the accounting voucher object, and then the relevant interface of the rule engine subsystem is called to transfer the accounting voucher object to the rule engine subsystem.

The second way is to process the historical transaction data of major business systems. Firstly, task scheduling plan must be set in task scheduling. The batch-running program that runs once every time adopts javax jms MessageListener technology. After a scheduled task is triggered at a certain point in time, the Messagemessage method of MessageListener will receive the information of this scheduled task. Therefore, the batch-running program that triggers the timed batch-running task directly goes to the database backup of the business system by adopting DBLlink technology between the management accounting system and the business system database. The rule engine subsystem is responsible for converting each accounting voucher into accounting entries, and recording the accounting vouchers and accounting entries into the database in turn.

## 4. Transformation of Financial Accounting under the Management Accounting System Based on Drools

With the rapid development of the company's business, relying on the accounting method of financial accounting can no longer meet the needs of the company's current accounting management. In order to achieve real-time accounting, Drools rule engine is introduced in this system so that the transaction records can automatically match accounting rules after passing through the rule engine subsystem, which has the following advantages to realize the transformation of accounting mode:

### 4.1. Advanced Technology

The efficiency of automatic accounting is high, and the probability of occurring error is very small. All that needed is to configure the correct entry generation rules in the rule management subsystem. The accounting entry generation rules set up double-entry accounting entries according to the information of transaction data such as transaction platform number, transaction type, payment gateway number, merchant number, etc., which not only realizes automation in accounting, but also in many aspects, such as the generation of trial balance daily-cut accounting statements that is conducive to the transformation from financial accounting to management accounting.

### 4.2. Reasonable Structure

This system adopts B/S(Browser/Server) architecture, without installing any client. Users only need a terminal that can be connected to the network to access the background management system of the rule management subsystem to manage the accounting system, set accounting rules and manage relevant basic data of the accounting system, or to view and download related financial statements. Compared with the financial accounting system, there is no need to install SqlServer and other related third-party components before running. The current management accounting system provides structural advantages for the transformation of accounting modes.

## 5. Conclusion

In order to conform to the development of the artificial intelligence, the financial management of modern enterprises needs to be actively based on the background of artificial intelligence management, and solve the problem of lag existing in the current financial management. In this paper, the strategy of transformation from financial accounting to management accounting is analyzed. By designing a management accounting system based on Drools rule engine to realize the transformation from financial accounting to management accounting under the background of artificial intelligence, the architecture of the management accounting system is specifically analyzed, including: the network architecture and software architecture. Then the implementation of the core subsystem related to Drools technology application is studied. The system can realize automation in many aspects such as the generation of trial balance and daily accounting statements, thus promoting the transformation from financial accounting to management accounting under artificial intelligence, and advancing the long-term sustainable development of enterprises and social economy.

## Figures and Tables

**Figure 1:** Structure of rule engine.

**Figure 2:** Structure of Rete rule matching algorithm.

**Figure 3:** Systematic network architecture.

**Figure 4:** System software architecture.

**Figure 5:** Saturn framework.

## Data Availability

All data generated or analysed during this study are included in this published article.
